RETRACTED

# The Investigation of Pulmonary Function Changes of COVID-19 Patients in Three Months

**DOI:** 10.1155/2022/9028835

**Published:** 2022-01-17

**Authors:** Lingyan Ye, Guifei Yao, Shuangxiang Lin, Yicheng Fang, Xi Chen, Liangxing Wang, Susu He

**Affiliations:** ^1^Department of Respiratory Medicine, Taizhou Hospital of Zhejiang Province Affiliated to Wenzhou Medical University, Linhai, Zhejiang, China; ^2^Department of Radiology, Taizhou Hospital of Zhejiang Province Affiliated to Wenzhou Medical University, Linhai, Zhejiang, China; ^3^Department of Respiratory Medicine, The First Affiliated Hospital of Wenzhou Medical University, Wenzhou, Zhejiang, China

## Abstract

**Background:**

Novel coronavirus disease 2019 (COVID-19) was discovered in December 2019 and has infected more than 80 million people worldwide, and more than 50 million people have achieved a clinical cure. In this study, the pulmonary function results of patients after clinical medicine for three months were reported.

**Objective:**

To investigate the effect of COVID-19 on lung function in patients.

**Methods:**

A retrospective analysis was performed on 56 COVID-19-infected patients who were cured after the clinical treatment at Taizhou Public Health Medical Center in Zhejiang Province from January 31, 2020, to March 10, 2020. At discharge and three months after discharge, lung function was measured, including inspiratory vital capacity (IVC), forced vital capacity (FVC), forced expiratory volume in first second (FEV1), forced expiratory volume in first second to inspiratory vital capacity (FEV1/IVC), maximum mid-expiratory flow rate (MEF), peak expiratory flow rate (PEF), and carbon monoxide dispersion (DLCO).

**Results:**

At discharge, there were 37 patients (66.1%) with pulmonary dysfunction, 22 patients (39.3%) with ventilation dysfunction, 31 cases (55.4%) with small airway dysfunction, and 16 cases (28.6%) with restricted ventilation dysfunction combined with small airway dysfunction. At 3 months after discharge, 24 of the 56 patients still had pulmonary dysfunction and all of them had small airway dysfunction, of which 10 patients (17.9%) were restricted ventilation dysfunction combined with small airway dysfunction. DLCO was measured three months after discharge. Twenty-nine patients (51.8%) had mild to moderate diffuse dysfunction. All pulmonary function indexes of 56 patients recovered gradually after 3 months after release, except FEV1/IVC, and the difference was statistically significant (*P* < 0.05). There were 41 patients of normal type (73.2%) and 15 patients of severe type (26.8%). Among the 15 severe patients, 8 patients (53.3%) had ventilation dysfunction at discharge, 9 patients (60%) had small airway dysfunction, 4 patients (26.7%) still had ventilation dysfunction 3 months after discharge, 7 patients (46.7%) had small airway dysfunction, and 10 patients (66.7%) had diffuse dysfunction. Among the 41 common type patients, 14 patients (34.1%) had ventilation dysfunction at discharge, 22 patients (53.7%) had small airway dysfunction, 6 patients (14.6%) still had ventilation dysfunction 3 months after discharge, 17 patients (41.5%) had small airway dysfunction, and 19 patients (46.3%) had diffuse dysfunction. Patients with severe COVID-19 had more pulmonary impairment and improved pulmonary function than normal patients.

RETRACTED

**Conclusion:**

COVID-19 infection can cause lung function impairment, manifested as restricted ventilation dysfunction, small airway dysfunction, and diffuse dysfunction. The pulmonary function of most patients was improved 3 months after clinical cure and discharge, and some patients remained with mild to moderate diffuse dysfunction and small airway dysfunction.

## 1. Introduction

Since December 2019, COVID-19, first discovered in Wuhan, has rapidly spread to many countries and regions worldwide, and is now a pandemic with high morbidity and mortality that has occurred all over the world [1, 2]. Severe acute respiratory syndrome coronavirus 2 (SARS-CoV-2) is a beta coronavirus. There have been two previous severe worldwide beta coronavirus infections: severe acute respiratory syndrome (SARS) and Middle East respiratory syndrome (MERS) [3, 4]. This kind of virus mainly leads to respiratory tract infection in humans, which can occur in patients with severe pneumonia, pulmonary edema, ARDS or multiple organ failure, and death, and lung dysfunction is a common complication [5].

There have been several recent literature reports [5–8], which indicate that most of the patients with COVID-19 mainly represented with fever, dry cough, and sputum in some patients. With the progress of the disease, some patients may show shortness of breath one week after onset. Prior study has reported [9] that, the infection of SARS, which is also one kind of beta coronavirus, can result in some patients with pulmonary fibrosis. Lung function impairment in survival patients is found in the clinical lung function follow-up, including obstructive ventilatory function, restrictive ventilatory function, and dispersion function obstacles [10, 11]. There is an obvious correlation between patients with residual lesions in the lung and lung function impairment [11].

At present, there are few reports on the recovery of lung function in COVID-19 patients after recovery. So will the infection of COVID-19 patients lead to impaired lung function or even left pulmonary fibrosis? Our study aims at elucidating the effect of novel COVID-19 infection on the lung function of patients and providing clues for the later pulmonary rehabilitation therapy of clinically cured patients with COVID-19.

RETRACTED

## 2. Methods

### 2.1. Patients

This study retrospectively collected 56 patients with COVID-19 who met the clinical cure criteria after hospitalization in Taizhou Public Health Center of Zhejiang Province from January 31, 2020, to March 10, 2020 [12]; that is, respiratory symptoms were significantly improved, two pharyngeal swabs for novel coronavirus nucleic acid tests were both negative, longer than 24 h, and lung CT showed significant absorption of lesions. The respiratory secretions obtained by nasopharyngeal swabs were detected by RT-PCR for novel coronavirus positive before admission, and the patients were diagnosed as COVID-19 according to the Chinese COVID-19 protocol [12]. The diagnostic criteria for patients with severe COVID-19 were as follows: (1) respiratory distress, respiratory rate (RR) > 30 times/min; (2) average oxygen saturation ≤93%, arterial oxygen partial pressure/oxygen concentration (PaO_2_/FiO_2_) ≤ 300; and (3) chest imaging lesion progression [13] within 24–48 hours > 50%. We collected the age, sex, and smoking history of the enrolled patients, and performed pulmonary function tests at discharge and follow-up three months after release. This study was approved by the Ethics Committee of Taizhou Hospital of Taizhou Medical Group (Center) of Zhejiang Province, and patients' written informed consent was obtained after retrospective data collection.

### 2.2. Lung Function Test

All patients were examined for pulmonary function after reaching clinical cure. The detection indexes included inspiratory vital capacity (IVC), forced vital capacity (FVC), forced expiratory volume in 1s (FEV1), and the ratio of forced expiratory volume in the first second to inhaled vital volume FEV1/IVC. The maximum expiratory flow at 25% of vital capacity is denoted by MEF 25, maximum expiratory flow at 50% of vital capacity is denoted by MEF 50, maximum expiratory flow at 75% of vital capacity is denoted by MEF 75, peak expiratory flow is denoted as PEF, and diffusion capacity for carbon monoxide is denoted as DLCO. All of the patients tested for lung function were seated comfortably in separate and enclosed rooms, and were tested for lung function three times, with the highest FEV1 value. Except FEV1/IVC and FEV1/FVC, other pulmonary function indexes were expressed as the percentage of measured values to predicted values. The lung function tester used in this study was Powercube Body BF lung function tester produced by Ganshorn Medizin Ectronic (Germany). All lung function tests were performed by the same technician. All practices are performed and assessed in accordance with the new standards issued by the European Respiratory Society/American Thoracic Society (ERS/ATS) in 2017 [14, 15]. Pulmonary function criteria include the following: (1) pulmonary ventilation function—FVC% <80%, FEV1% < 80%, FEV1/FVC > 70%, indicating restrictive ventilation dysfunction; FVC% >80%, FEV1% < 80%, and FEV1/FVC < 70% were obstructive ventilation dysfunction. The degree of pulmonary ventilation dysfunction was expressed by FEV1%, which was divided into mild damage (≥70%), moderate damage (50% ≤ FEV1% < 70%), severe damage (35% ≤ FEV1% < 50%), and very severe damage (<35%) [15, 16]; (2) pulmonary diffusion function—DLCO% ≥ 80% was normal, mild disorder (60% ≤DLCO% < 80%), moderate disorder (40% ≤ DLCO % < 60%), and severe disorder (DLCO% < 40%) [14, 15]; And (3) small airway function—MEF25%, MEF 50% ≥ 70% is normal, mild impairment (60% ≤ MEF25%, MEF 50% < 70%), moderate impairment (40% ≤ MEF25%, MEF 50% < 60%), and severe impairment (MEF25%, MEF 50% < 40%) [15].

RETRACTED

### 2.3. Statistical Analysis

All statistical analyses were carried out using SPSS (v20.0). Categorical variables were described as frequency rates and percentages, and continuous variables were described using mean and median.

## 3. Results

The median age of 56 patients was 44.13 ± 10.15 years (range, 23–79 years old), and 50 percent of them were male; 4 patients (7.14%) had a history of smoking; and 2 patients (3.57%) had a history of COPD (chronic obstructive pulmonary disease). There were 41 patients of normal type (73.2%) and 15 patients of severe type (26.8%) (Table 1).

At discharge, 37 (66.1%) of the 56 COVID-19 patients had pulmonary dysfunction: 22 (39.3%) showed ventilation dysfunction, including 15 (26.8%) with mild and 7 (12.5%) with moderate, 1 (1.8%) with obstructive ventilation dysfunction, and 21 (37.5%) with restrictive ventilation dysfunction. Thirty-one patients (55.4%) presented small airway dysfunction, of which 16 patients (28.6%) were restricted ventilation dysfunction combined with small airway dysfunction. Three months after discharge, 24 patients (42.9%) remained with pulmonary dysfunction, all of which were presented as small airway dysfunction, and 10 patients (17.9%) were restricted ventilation dysfunction combined with small airway dysfunction. Fifty-six patients with COVID-19 were tested by DLCO 3 months after cure and discharge, 29 patients (51.8%) had diffuse dysfunction, 10 patients (17.9%) had restricted ventilation dysfunction and small airway dysfunction, of which 23 patients (41.1%) had mild diffuse dysfunction, and 6 patients (10.7%) had moderate diffuse dysfunction (Table 2). Lung function indexes of 56 patients at discharge such as IVC, FEV1, FVC, MEF 25, MEF 50, MEF 75, and PEF were 62.5 ± 14.4, 83.4 ± 12.3, 84.8 ± 12.9, 71.1 ± 37.6, 79.6 ± 25.1, 87.3 ± 18.7, and 85.2 ± 18.6, respectively, and three months after discharge, indexes improved to 83.1 ± 19.0, 92.7 ± 15.0, 92.9 ± 12.8, 78.6 ± 34.8, 92.0 ± 31.0, 101 ± 22.4, and 102 ± 18.6. So the pulmonary function indexes of 56 patients (IVC, FEV1, FVC, MEF 25, MEF 50, MEF 75, PEF) changed significantly on the day of discharge and 3 months after discharge, and the difference was statistically significant (*P* < 0.05) (as shown in Table 3), which indicated that the pulmonary function impairment of COVID-19 patients was gradually recovered 3 months after discharge compared with that at discharge, and the pulmonary function of most patients had basically returned to normal. The decreasing trend of FEV1/IVC may be related to the faster recovery rate of IVC than that of FEV1 over time.

RETRACTED

Pulmonary function in mild and severe COVID-19 patients: Among the 15 severe patients, 8 patients (53.3%) had ventilation dysfunction at discharge, 9 patients (60%) had small airway dysfunction, 4 patients (26.7%) still had ventilation dysfunction 3 months after discharge, 7 patients (46.7%) had small airway dysfunction, and 10 patients (66.7%) had diffuse dysfunction. Among the 41 common type patients, 14 patients (34.1%) had ventilation dysfunction at discharge, 22 patients (53.7%) had small airway dysfunction, 6 patients (14.6%) still had ventilation dysfunction 3 months after discharge, 17 patients (41.5%) had small airway dysfunction, and 19 patients (46.3%) had diffuse dysfunction (Table 2). Lung function injury is more typical in severe patients than in common patients. Three months after clinical cure and discharge, lung function in light and severe patients all recovered well, and the improvement in IVC and MEF25 indexes in severe patients was more obvious (Table 4).

## 4. Discussion

Novel coronavirus has spread around the world and seriously threatened people's safety and health. The pandemic of COVID-19 has posed a significant challenge to the global health service system. The coronavirus is high transmissible with strong pathogenicity, transmitted by respiratory droplets or close contact. With the invasion of the coronavirus in the respiratory tract, the patient could have lung tissue injured directly or get an acute respiratory distress syndrome incurred by the inflammatory immune response, which has a high fatality rate [17, 18]. Even after the clinical cure, there are still patients whose chest CT lesions are not fully absorbed, with remaining pulmonary interstitial changes and the lung function damage, thus affecting the life quality of these patients [19]. Recent studies have shown that COVID-19 survivors may have long-term pulmonary dysfunction [20].

RETRACTED

The sequela of some SARS patients is pulmonary fibrosis [9]. Recent studies have shown that the pathological features of COVID-19 are similar to those of SARS. Interstitial mononuclear inflammatory infiltration and alveolar septal fibroblast proliferation can also be found in the lungs of COVID-19 patients [21]. In this study, lung function detection was performed on 56 cured patients on the day of discharge. It showed that 66.1% of the patients had lung function impairment, which was mild and moderate pulmonary dysfunction, and no severe or extremely severe pulmonary dysfunction was observed. The pathophysiological changes after COVID-19 infection mainly were double diffuse lung tissue damage associated with cellular fiber mucous exudate, leading to a wide range of interstitial inflammatory change [22], whose manifestations after the invasion of the coronavirus in the airway were bronchial epithelial basement membrane thickening, alveolar walls transparent sample, structure of lung tissue damage, extracellular matrix accumulation in great quantities, interstitial fibrosis caused by the inflammation injury of lung tissue, interstitial fibrosis II type alveolar epithelial injury at the same time, and the lack of surface active substance, which leads to the closed small airways, and these pathological changes result in the decrease of lung compliance and abnormal small airway function, thereby seriously affecting pulmonary gas exchange. The final manifestations were restricted ventilation dysfunction, small airway dysfunction, and diffuse dysfunction [23]. The study results of Wang et al. [24] showed that residual lung injury and lung function impairment in patients with mild symptoms of COVID-19 could last for longer than one month. The pulmonary function results of this study showed that 21 patients (37.5%) met FVC% < 80%, FEV1% < 80%, and FEV1/FVC > 70% and had restricted ventilation dysfunction at discharge; and 31 patients (55.4%) had MEF 25 and MEF 50 < 70% predictive value, and had small airway dysfunction. Three months after discharge, 24 patients (42.9%) still had small airway dysfunction, and 10 of them (17.9%) had restricted ventilation dysfunction. The above results were consistent with pathological changes. The results in Table 4 of this study showed that the indexes of IVC, FEV1, FVC, MEF25, and MEF50 in severe patients were lower than those in normal type patients at discharge. The proportion of severe ventilation dysfunction and small airway dysfunction in severe patients at discharge and three months after discharge was also higher than that in normal type patients, suggesting that lung function injury in severe patients was more common than that in normal type patients. Previous results reported from a series of hospitalized COVID-19 patients showed that impaired lung diffusion function (TLCO <80% prediction) was the most common manifestation, in which obvious lung function deficit was only about one-tenth [25]. At 3 months after discharge, the mean value of DLCO% in 56 patients was (84.8% ± 19.2%), and 29 patients (51.8%) had DLCO% < 80%. Diffuse dysfunction was represented, including 23 patients with mild disorder and 6 patients with moderate disorder. Diffuse dysfunction was more common in severe COVID-19 patients (66.7%).

RETRACTED

Our research shows that reaction ventilation dysfunction and pulmonary function index of small airway dysfunction IVC, FEV1 and FVC, MEF 25, and MEF 50 recover gradually over time. The lung function of 57% patients recovers well at three months after cured and discharge, which is consistent with a recent study about the lung injury recovery status of the the SARS patients after 15 years [26]. Therefore, we can preliminarily infer that the lung function of COVID-19 patients, especially FEV1, FVC, MEF25, and MEF50, could recover gradually over time, suggesting that the interstitial inflammatory changes and interstitial fibrosis caused by or secondary to COVID-19 could be slowly recovered instead of progressive development. Unfortunately, we did not conduct the DLCO test at the time of discharge, so we could not evaluate the recovery of diffusion function. Our research results also show that the lung function damage in severe patients is more serious, with more apparent improvements in IVC (84.9 ± 19.8) and MEF25 indicators (80.2 ± 38.2) compared with that in normal type patients (IVC (82.4 ± 18.9) and MEF25 (78.0 ± 33.8)), indicating that with effective early management for heavy COVID-19 patients, the lung function could get better improvement. In combination with our study, some patients with COVID-19 have mild to moderate impairment in small airway or diffuse function on the day of release and 3 months after discharge, suggesting that the pulmonary function of COVID-19 patients has not been fully recovered in the early stage of rehabilitation. Combined with their pulmonary pathological changes, it is not still clear whether it is related to pulmonary interstitial lesions or pulmonary fibrosis lesions, which we will leave in our future study.

Because the detection of lung function is safe, noninvasive, and easy to be accepted by patients, it can be used as an objective indicator for clinical monitoring and evaluation of the pulmonary outcome of COVID-19 patients during recovery. This study shows that COVID-19 patients have pulmonary function impairment after clinical cure and discharge, mainly in dispersion dysfunction and small airway dysfunction. The pulmonary function could be improved gradually over time, and early pulmonary rehabilitation intervention might be helpful to the recovery of pulmonary function.

RETRACTED

## Figures and Tables

**Table 1:** Characteristics of the patients infected with COVID-19 (*n* = 56).

Characteristic	Results
*Age (years)*	
Median	44.13 ± 10.15
Range	23–79
<30	3 (5.4%)
30–49	35 (62.5%)
50–69	16 (28.6%)
>70	2 (3.5%)
*Sex*	
Men	28 (50%)
Women	28 (50%)
Smoking history	4 (7.14%)
Chronic obstructive pulmonary disease	2 (3.57%)
*Type*	
Severe	15 (26.8%)
Nonsevere	41 (73.2%)

Data are *n* (%), *n*/*N* (%), and median.

**Table 2:** Pulmonary function characteristics of COVID-19 patients.

Pulmonary dysfunction	On the day of discharge			Three months after discharge		
	All (*N* = 56)	Severe (*N* = 15)	Nonsevere (*N* = 41)	All (*N* = 56)	Severe (*N* = 15)	Nonsevere (*N* = 41)
Ventilation dysfunction	22 (39.3%)	8 (53.3%)	14 (34.1%)	10 (17.9%)	4 (26.7%)	6 (14.6%)
Mild ventilation dysfunction	15 (26.8%)	5 (33.3%)	10 (24.4%)	5 (8.9%)	2 (13.3%)	3 (7.3%)
Moderate ventilation dysfunction	7 (12.5%)	3 (20%)	4 (9.7%)	5 (8.9%)	2 (13.3%)	33 (7.3%)
Small airway dysfunction	31 (55.4%)	9 (60%)	22 (53.7%)	24 (42.9%)	7 (46.7%)	17 (41.5%）
Ventilation dysfunction with small airway dysfunction	16 (28.6%)	6 (40%)	10 (24.4%)	10 (17.9%)	4 (26.7%)	6 (14.6%)
Disseminated dysfunction				29 (51.8%)	10 (66.7%)	19 (46.3%)

**Table 3:** Pulmonary function changes of patients infected with COVID-19.

Pulmonary function (%Pred)	On the day of discharge (*N* = 56)	Three months after discharge (*N* = 56)	*P* value
IVC	62.5 ± 14.4	83.1 ± 19.0	<0.001
FVCex	84.8 ± 12.9	92.9 ± 12.8	0.00115
FEV1	83.4 ± 12.3	92.7 ± 15.0	<0.001
MEF25	71.1 ± 37.6	78.6 ± 34.8	0.0275
MEF50	79.6 ± 25.1	92.0 ± 31.0	0.0222
MEF75	87.3 ± 18.7	101 ± 22.4	<0.001
PEF	85.2 ± 18.6	102 ± 18.6	<0.001
DLCO		84.8 ± 19.2	

**Table 4:** Pulmonary function changes in patients with different types of COVID-19.

Pulmonary function (%Pred)	On the day of discharge			Three months after discharge		
	Nonsevere (*N* = 41)	Severe (*N* = 15)	*P* value	Nonsevere (*N* = 41)	Severe (*N* = 15)	*P* value
FEV1/IVC	112 ± 21.5	114 ± 21.7	0.854	92.4 ± 20.7	82.1 ± 6.71	0.007
IVC	64.4 ± 13.8	57.7 ± 15.2	0.135	82.4 ± 18.9	84.9 ± 19.8	0.689
FVCex	86.9 ± 11.6	79.6 ± 14.9	0.096	94.6 ± 11.8	88.9 ± 14.5	0.176
FEV1	85.3 ± 11.9	78.8 ± 12.5	0.0856	94.0 ± 14.2	89.6 ± 16.9	0.367
MEF25	73.7 ± 41.1	64.6 ± 26.7	0.336	78.0 ± 33.8	80.2 ± 38.2	0.841
MEF50	81.4 ± 26.0	75.3 ± 23.0	0.394	92.8 ± 29.7	89.9 ± 35.1	0.769
MEF75	86.3 ± 17.1	89.6 ± 22.6	0.61	100 ± 20.1	102 ± 27.9	0.79
PEF	82.5 ± 17.7	92.0 ± 19.6	0.105	101 ± 17.9	105 ± 20.5	0.455
DLCO				87.9 ± 16.9	79.6 ± 22.4	0.209

RETRACTED

## Data Availability

Data are available upon request from the corresponding author.
